The article "LncRNA CARMN Affects Hepatocellular Carcinoma Prognosis by Regulating the miR-192-5p/LOXL2 Axis" was published in 2022. Journal: Oxid Med Cell Longev.

# LncRNA CARMN Affects Hepatocellular Carcinoma Prognosis by Regulating the miR-192-5p/LOXL2 Axis

**DOI:** 10.1155/2022/9277360

**Published:** 2022-10-08

**Authors:** Xiaokang Wang, Shulong Wu, Yi Yang, Jingjing Zhao

**Affiliations:** ^1^Department of Pharmacy, Shenzhen Longhua District Central Hospital, Shenzhen, China; ^2^Guangdong Provincial Key Laboratory of Research and Development of Natural Drugs, and School of Pharmacy, Guangdong Medical University, Dongguan, China; ^3^The Marine Biomedical Research Institute of Guangdong Zhanjiang, Zhanjiang, China; ^4^Department of Pharmacy, South China Hospital of Shenzhen University, Shenzhen, China; ^5^Health Science Center, Shenzhen University, Shenzhen, China; ^6^Department of Pharmacy, Guangdong Women and Children Hospital, Guangzhou, China

## Abstract

**Background:**

Hepatocellular carcinoma (HCC) is aggressive cancer with a poor prognosis. It has been suggested that the aberrant expression of LOXL2 is associated with the development of HCC, but the exact mechanism remains unclear. This research is aimed at examining the expression level and prognostic value of LOXL2 in hepatocellular carcinoma and its relationship with immune infiltration and at predicting its upstream noncoding RNAs (ncRNAs).

**Method:**

The transcriptome data of HCC was first downloaded from The Cancer Genome Atlas (TCGA) database to investigate the expression and prognosis of LOXL2. Then, the starBase database was used to find the upstream ncRNAs of LOXL2, and correlation analysis and expression analysis were performed. Finally, the Tumor Immune Estimation Resource (TIMER) was used to explore the association between LOXL2 and immune cell infiltration.

**Result:**

CARMN was considered to be the potential upstream lncRNA for the hsa-miR-192-5p/LOXL2 axis in HCC. Furthermore, the level LOXL2 was markedly positively associated with tumor immune cell infiltration and immune checkpoint expression in HCC.

**Conclusion:**

Higher expression of LOXL2 mediated by microRNA (miRNA) and long noncoding RNAs (lncRNA) is associated with poor overall survival (OS), immune infiltration, and immune checkpoint expression in HCC.

## 1. Introduction

Hepatocellular carcinoma (HCC) is the main type of liver cancer (LC). As the sixth most common cancer in the world, it is the second largest cause of cancer-related death and the most common primary liver cancer with poor prognosis [1, 2]. The morbidity and mortality rates of HCC are expected to significantly increase in the next few years [2]. Epidemiological data show that hepatitis virus infection [3], aflatoxin [4], type 2 diabetes [5], alcohol consumption [6], and smoking [7] are all predisposing factors for liver cancer. Despite remarkable improvements in the diagnosis and treatment of HCC, such as surgical resection [8] and sorafenib-regorafenib sequential therapy [9], patients with HCC often exhibit local invasion and metastasis resulting in a poor overall survival (OS) rate [10, 11]. Therefore, early screening and diagnosis of HCC are particularly crucial, and there is an urgent need to find specific and sensitive biomarkers.

The article "LncRNA CARMN Affects Hepatocellular Carcinoma Prognosis by Regulating the miR-192-5p/LOXL2 Axis" was published in 2022. Journal: Oxid Med Cell Longev.

Lysyl oxidase (LOX), an extracellular enzyme, plays a key role in the covalent cross-linking of collagen fibers by oxidizing deamino-specific lysine and hydroxylysine in the telopeptide structural domain of the collagen molecule to form allantoin [12]. In addition to LOX, there are four other members in the lox protein family, namely, LOX-like proteins (LOXL1, LOXL2, LOXL3, and LOXL4) [13, 14]. Among these proteins, LOXL2 is considered to be an important regulator of tumor progression, and previous studies reported that LOXL2 is significantly overexpressed in human HCC tissues compared to nontumor tissues [15]. Studies demonstrated that elevated levels of LOXL2 might contribute to tumor progression and metastasis by promoting tumor cell invasion and remodeling of the tumor microenvironment [16, 17]. Considering the major role of LOXL2, we further investigated the role of LOXL2 in the development of HCC progression based on previous studies.

In this study, the expression level of the LOXL2 and its relationship with prognosis were first analyzed in various common cancers. Next, we found some noncoding RNAs (microRNAs (miRNAs)) and long noncoding RNAs (lncRNAs) as regulatory molecules of LOXL2 by bioinformatics analysis, so as to establish the LncRNA-miRNA-mRNA regulatory network and explore the mechanism of HCC at a deeper level. Moreover, the correlation of LOXL2 expression with immune cell infiltration, biomarkers of immune cells and immune checkpoints was finally discussed.

## 2. Methods

### 2.1. Download, Process, and Analysis of The Cancer Genome Atlas (TCGA) Data

The Cancer Genome Atlas (TCGA) database (https://portal.gdc.cancer. gov/) is a collaboration between the National Cancer Institute (NCI) and the National Human Genome Research Institute (NHGRI) for cancer research. It provides a large and free reference for cancer research by collecting and organizing various cancer-related histological data. A total of 33 cancer types are currently included. Data in this research was obtained from the Liver Hepatocellular Carcinoma (LIHC) cohort, and then Log2 transformed. The expression levels of LOXL2 in tumor tissues were compared with normal tissues using Wilcoxon rank sum test in the eighteen cancers (BLCA, BRCA, CHOL, COAD, ESCA, GBM, HNSC, KICH, KIRC, KIRP, LIHC, LUAD, LUSC, PRAD, READ, STAD, THCA, and UCEC), and then visualized by box plots. The analysis was performed using the R software “limma” and “ggplot2” packages [18].

The article "LncRNA CARMN Affects Hepatocellular Carcinoma Prognosis by Regulating the miR-192-5p/LOXL2 Axis" was published in 2022. Journal: Oxid Med Cell Longev.

### 2.2. Analysis of LOXL2 Expression and Prognosis in Pan-Cancer by GEPIA Database

The GEPIA database (http://gepia.cancer-pku.cn/) integrates TCGA cancer data with GTEx normal tissue data, exploiting bioinformatics techniques to drill down into novel cancer targets and markers. In this research, we analyzed the expression LOXL2 in tumor and normal samples and prognosis in pan-cancer by the GEPIA database [19]. The boxplots and Kaplan–Meier plots were downloaded for visualizing the results of differential expression analysis and survival analysis.

### 2.3. Prediction and Analysis of Upstream miRNAs of LOXL2

The starBase database (https://starbase.sysu.edu.cn/) is used to analyze data related to multiple cancers integrated from the TCGA project. It provides a platform for predicting miRNA targets by searching for miRNA targets through high-throughput CLIP-Seq experimental data and degradome experimental data which include lncRNAs, miRNAs, snoRNAs, and mRNAs [20]. We use this platform to detect the upstream miRNA of LOXL2 in this research. After searching with the keyword “LOXL2” in “Target Gene” module and selecting the “miRNA-mRNA” option, the upstream miRNAs that LOXL2 may bind to would be presented. The filtering condition for screening is that the miRNAs would be predicted in two or more programs. The regulatory network between these predicted miRNAs and LOXL2 was demonstrated with Cytoscape software [21]. Among them, miRNAs with correlation coefficients greater than 0.2 were included in the subsequent analysis. In addition, expression analysis for the selected miRNA was also performed.

### 2.4. Prediction and Analysis of Upstream lncRNAs of miRNA

The upstream lncRNA of the miRNAs selected in the prior step was also identified in starBase database [20]. It has been known that miRNAs can bind to target mRNAs and inhibit their translation or cause mRNA degradation to achieve the function of posttranscriptional regulation of gene expression. The ceRNA theory represents a new model of gene expression regulation. ceRNA molecules (lncRNA, circRNA, etc.) can compete to bind the same miRNA through miRNA Response Element (MRE) to regulate each other's expression levels [22–24]. Therefore, the eligible lncRNA should be negatively correlated with miRNA and positively correlated with mRNA.

### 2.5. Analysis of Immune Infiltration in HCC

The TIMER database (https://cistrome.shinyapps.io/timer/) is a comprehensive resource for the systematic analysis of immune infiltrates in diverse cancer types [25]. TIMER database is used to detect six types of immune cell (including dendritic cells, macrophages, neutrophils, CD4+ T cells, CD8+ T cells, and B cells) infiltration in tumor tissues with RNA-Seq expression profiling data. In this study, the TIMER database was used to estimate the correlation between LOXL2 and the extent of infiltration of specific immune cell subpopulations. Additionally, considering the potential oncogenic role of LOXL2 in HCC, the relationship of LOXL2 with immune checkpoints (involving CTLA4/PDCD1/CD274) was assessed as well.

The article "LncRNA CARMN Affects Hepatocellular Carcinoma Prognosis by Regulating the miR-192-5p/LOXL2 Axis" was published in 2022. Journal: Oxid Med Cell Longev.

### 2.6. Statistical Analysis

The statistical analysis was automatically calculated by the online database or statistical software. *p* value less than 0.05 was considered statistically significant.

## 3. Result

### 3.1. The Expression Level of LOXL2 in Pan-Cancers

To explore the role of LOXL2 in the development of HCC progression, we first analyzed the expression level of LOXL2 in 18 types of cancer based on the TCGA database, which found that LOXL2 was markedly upregulated in 16 cancer types, including BLCA, BRCA, CHOL, COAD, ESCA, GBM, HNSC, KIRC, KIRP, LIHC, LUAD, LUSC, READ, STAD, THCA, and UCEC and was significantly downregulated in PRAD. However, there was no significant difference between KICH and normal tissues (Figure 1(a)). Next, to further confirm this result, the GEPIA database was also used to evaluate the LOXL2 expression levels in these cancers. As presented in Figure 1(b), LOXL2 was significantly increased in CHOL, ESCA, GBM, HNSC, KIRC, LIHC, and STAD, whereas it was decreased in PRAD, compared with normal tissues. Also, no statistically significant difference was observed in BLCA, BRCA, COAD, KICH, KIRP, LUAD, LUSC, READ, THCA, and UCEC (Figures 1(c)–1(s)). Taken together, LOXL2 was upregulated in CHOL, ESCA, GBM, HNSC, KIRC, LIHC, and STAD and downregulated in PRAD, which indicated that LOXL2 was in connection with the development of the above cancer types.

### 3.2. The Prognostic Value of LOXL2 in Pan-Cancers

GEPIA platform was used to analyze the prognostic value of LOXL2 in pan-cancers, and OS is selected to be the outcome indicator. As shown in Figure 2, higher expression of LOXL2 was associated with worse OS in LIHC, LUAD, and LUSC. Consequently, combining the expression of LOXL2 between tumor and normal tissues and its prognostic value, LOXL2 may be utilized as an unfavorable prognostic biomarker in patients with LIHC.

### 3.3. Further Exploration of LOXL2 Expression Levels and Survival Conditions in HCC

The expression analyses of LOXL2 in unpaired samples, paired samples, and different clinical subgroups are shown in Figure 3. With the increased expression level of LOXL2, the pathologic stage of HCC increases accordingly. Also, we found that in female, the expression level of LOXL2 was higher than that in male.  Table 1 listed the LOXL2 expression data and clinical data for 374 HCC patients. We observed a significant association between LOXL2 expression and clinicopathological features, such as gender, T stage, and histologic grade (*p* < 0.05).

The article "LncRNA CARMN Affects Hepatocellular Carcinoma Prognosis by Regulating the miR-192-5p/LOXL2 Axis" was published in 2022. Journal: Oxid Med Cell Longev.

As for survival, we further performed subgroup analyses to assess the impact of LOXL2 expression on OS of patients with HCC according to age, gender, pathological stage, and differentiation grade. We found that high-expression of LOXL2 resulted in poor survival in patients older than 60 years old and in male patients (Figure 4).

### 3.4. Prediction and Analysis of Upstream miRNA of LOXL2

MiRNAs represent a class of noncoding single-stranded RNA molecules of approximately 22 nucleotides in length encoded by endogenous genes, which are involved in the posttranscriptional regulation of gene expression. Twenty-two possible miRNAs were found in the starBase database according to the rules, and the regulatory network was presented in Figure 5(a). Notably, the miRNA that regulates the mRNA must be negatively correlated with that mRNA. Therefore, the screening criteria were set: the value of the correlation coefficient was less than -2 and the *p* value was less than 0.05. Finally, only hsa−miR−192−5p met the conditions (Figure 5(b)). Furthermore, hsa−miR−192−5p was found to be lowly expressed in HCC tissues and patients with lower hsa−miR−192−5p expression had a better prognosis. (Figures 5(c) and 5(d)).

### 3.5. Prediction and Analysis of Upstream lncRNAs of Hsa−miR−192−5p

Also, the upstream lncRNAs of miRNAs can be searched in the starBase database. After downloading the twelve relevant lncRNAs from the database, the regulatory network was visualized using Cytoscape software (Figure 6(a)). However, among these lncRNAs, only CARMN was negatively correlated with hsa−miR−192−5p (*R* < −2, *P* < 0.05) and positively correlated with LOXL2 (*R* > 2, *P* < 0.05) (Figures 6(b) and 6(c)). Besides, expression analysis showed that CARMN was highly expressed in the tumor samples (Figure 6(d)). Thus, CARMN was selected as a promising upstream lncRNA for the miR-192-5p/LOXL2 axis in HCC.

### 3.6. LOXL2 Correlates with Immune Cell Infiltration in HCC

The relationship between LOXL2 and immune cell infiltration was investigated using the timer database because the level of immune cells is associated with the proliferation and development of tumor cells.

The expression of LOXL2 was positively correlated with the infiltration of dendritic cells, neutrophils, macrophages, CD8+ T cells, CD4+ T cells, and B cells (Figure 7). Among them, CD4+ T Cells, macrophages, and neutrophils showed the strongest positive correlation.

The article "LncRNA CARMN Affects Hepatocellular Carcinoma Prognosis by Regulating the miR-192-5p/LOXL2 Axis" was published in 2022. Journal: Oxid Med Cell Longev.

### 3.7. The Relationship between LOXL2 and Immune Checkpoints in HCC

CD274, PDCD1, and CTLA-4 were known as critical immune checkpoints that are associated with immune escape in cancers. So, the relationship between LOXL2 and these checkpoints was analyzed via online tools. Both TIMER data analysis and GEPIA data analysis found a significant positive correlation of LOXL2 with CD274, PDCD1, and CTLA-4 (Figures 8(a)–8(f)).

## 4. Discussion

HCC is one of the most common malignant tumors in the world, and with the continuous development of medical technology and research on the molecular biology of tumors, targeted therapy for hepatocellular carcinoma is developing rapidly [1, 2]. TERT, MLL4, CCNE1, TP53, and CTNNB1 were identified as commonly mutated genes in HCC [26–30]. Despite the availability of many potential therapeutic targets, the incidence and mortality rates of patients with HCC are still increasing currently [8–11]. The overall survival rate remains suboptimal, so it is crucial to explore the underlying molecular mechanisms and oncogenes to provide new ideas for the diagnosis and treatment of HCC. Previous studies had uncovered the value of LOXL2 in different tumors, but the exact mechanism remains unclear [15, 31–33]. In this study, we discussed the role of LOXL2 in HCC through bioinformatics analysis to further understand the potential value of LOXL2.

In this present study, the expression of LOXL2 in various cancers was analyzed using different databases (TCGA database and GEPIA database), and it was concluded that LOXL2 was significantly differentially expressed in HCC. The next survival analysis using GEPIA online tool revealed that LOXL2 overexpression leads to a poorer prognosis in patients with HCC. Wu et al. constructed LOXL2-small interfering RNA using a lentiviral vector and investigated the effect of LOXL2 on the proliferation of HCC cell lines by reverse transcription-quantitative polymerase chain reaction and other experimental methods [34]. The results showed that LOXL2 was highly expressed in HCC tissues and that LOXL2 silencing reduced cell number, proliferation, colony formation, and cell growth, induced cell cycle arrest, and increased apoptosis [34]. This study and our results both demonstrated the oncogenic role of LOXL2 in HCC.

The starBase database contains seven programs that can be used to predict miRNAs, including TargetScan, miRmap, miRanda, PicTar, RNA22, PITA, and microT. Through these programs, twenty-two potential miRNAs were found for LOXL2. Among all these 22 possible miRNAs, only hsa-miR-192-5p showed a significant negative correlation with LOXL2. Subsequently, the data of miRNAs were downloaded from the TCGA database, and the differential analysis showed that hsa-miR-192-5p was lowly expressed in the tumor samples, and its low-expression was related to the poor prognosis of HCC. During the past decade, more and more studies are focusing on the role of miR-192-5p in cancers. For example, in Wang et al.'s experiment, they found that miR-192-5p-modified tumor-associated macrophages-derived exosome suppressed endometrial cancer progression by targeting IRAK1/NF-*κ*B signaling [35]. The role of miR-192-5p in HCC is also noteworthy. Previous studies revealed that miR-192-5p loss enhanced glycolysis and over produced lactate might further increase HCC malignant features via interacting with environmental nontumor cells [36]. Previous findings are consistent with our predictions. To summarize, hsa-mir-192-5p was found to be a vital regulatory molecule of LOXL2 in HCC.

The article "LncRNA CARMN Affects Hepatocellular Carcinoma Prognosis by Regulating the miR-192-5p/LOXL2 Axis" was published in 2022. Journal: Oxid Med Cell Longev.

According to the ceRNA theory, it is known that ceRNA inhibits the inhibitory effect of miRNA on mRNA by binding to it. Therefore, it is essential to find the upstream lncRNA of hsa-mir-192-5p because it plays a role in cancer development. StarBase bioinformatics software predictions showed that CARMN may be the upstream lncRNA of miR-192-5p. The expression analysis also showed that CARMN was highly expressed in the tumor samples. There is a paucity of research on CARMN in cancers. Sheng et al. found that overexpression of CARMN can promote the prognosis and chemosensitivity in breast cancer [37]. Other reports on the role of lncRNA CARMN in cancers are currently scarce. However, the results of this paper suggested that CARMN might influence the progression of HCC by regulating the miR-192-5p/LOXL2 axis.

The tumor microenvironment is a hot topic of research in recent years. The immune microenvironment, consisting of tumor-infiltrating lymphocytes (B cells, T cells) and other immune cells (such as dendritic cells, macrophages, and neutrophils), is an important part of the tumor microenvironment and is considered as the “seventh hallmark feature” of tumors, so more research is urgently needed to focus on the link between immune cell infiltration and tumors [38–40]. In our research, a positive correlation between LOXL2 expression and dendritic cells, neutrophils, macrophages, CD8+ T cells, CD4+ T cells, and B cell in HCC was observed. In addition, the correlation between LOXL2 expression and immune checkpoint markers (CD274, PDCD1, and CTLA-4) suggested a role for LOXL2 in immune regulation of tumor immunity. Consequently, it is hypothesized that tumor immune infiltration exerts an influential role in LOXL2-mediated HCC development.

The article "LncRNA CARMN Affects Hepatocellular Carcinoma Prognosis by Regulating the miR-192-5p/LOXL2 Axis" was published in 2022. Journal: Oxid Med Cell Longev.

The limitation of this study should be mentioned. First, this is a bioinformatics study based on an online database that lacks experimental validation. Second, in identifying CARMN as a potential upstream LncRNA for hsa-miR-192-5p in HCC, serval extreme values may leverage the true correlation and may lead to overestimation of the correlation of CARMN with hsa-miR-192-5p. Third, the results need to be interpreted carefully because many of the data do not have high-correlation values.

In short, CARMN was identified as a possible upstream lncRNA for miR-192-5p, which affects LOXL2 expression and promotes the progression of HCC. Our study suggests that LOXL2 may exert its tumorigenic effects by potentiating tumor immune cell infiltration and immune checkpoint expression. However, in the future, more relevant studies are still needed to verify these predictions by bioinformatics.

## Figures and Tables

**Figure 1:** Expression analysis for LOXL2 in multiple cancers. (a) The expression of LOXL2 in 18 types of human cancer based on TCGA cancer and normal data. (b)–(m) LOXL2 expression in GEPIA database. BLCA (b), BRCA (c), CHOL (d), COAD (e), ESCA (f), GBM (g), HNSC (h), KICH (i), KIRC (j), KIRP (k), LIHC (l), LUAD (m), LUSC (n), PRAD (o), READ (p), STAD (q), THCA (r), and UCEC (s) tissues compared with corresponding TCGA and GTEx normal tissues. ^∗^*p* value < 0.05, ^∗∗^*p* value < 0.01, ^∗∗∗^*p* value < 0.001.

**Figure 2:** The overall survival (OS) analysis for LOXL2 in various human cancers determined by the GEPIA database. (a)–(l) The OS plot of LOXL2 in BLCA (a), BRCA (b), CHOL (c), COAD (d), ESCA (e), GBM (f), HNSC (g), KICH (h), KIRC (i), KIRP (j), LIHC (k), LUAD (l), LUSC (m), PRAD (n), READ (o), STAD (p), THCA (q), and UCEC (r).

**Figure 3:** (a) Expression analysis for LOXL2 in unpaired sample. (b) Expression analysis for LOXL2 in paired sample. (c)–(f) Expression of LOXL2 in different clinical subgroups.

**Figure 4:** Subgroup Kaplan–Meier curve analysis for different clinicopathological factors.

**Figure 5:** Identification of hsa−miR−192−5p as a potential upstream miRNA of LOXL2 in HCC. (a) The miRNA-LOXL2 regulatory network. (b) The correlation between hsa−miR−192−5p and LOXL2 in HCC. (c) The expression of hsa−miR−192−5p in HCC and control normal samples. (d) The prognostic value of hsa−miR−192−5p in HCC.

**Figure 6:** Identification of CARMN as a potential upstream LncRNA of hsa−miR−192−5p in HCC. (a) The LncRNA- hsa−miR−192−5p regulatory network. (b) The expression correlation between hsa−miR−192−5p and CARMN in HCC. (c) The correlation between LOXL2 and CARMN in HCC. (d) The expression of CARMN in HCC and control normal samples.

The article "LncRNA CARMN Affects Hepatocellular Carcinoma Prognosis by Regulating the miR-192-5p/LOXL2 Axis" was published in 2022. Journal: Oxid Med Cell Longev.

**Figure 7:** The correlation of LOXL2 expression level with B cell, CD8+ T cell, CD4+ T cell, macrophage, neutrophil, or dendritic cell infiltration level in HCC.

**Figure 8:** Correlation of LOXL2 expression with CD274, PDCD1, and CTLA-4 expression in HCC (a) Spearman correlation of LOXL2 with expression of CD274 in HCC adjusted by purity using TIMER. (b) Spearman correlation of LOXL2 with expression of PDCD1 in HCC adjusted by purity using TIMER. (c) Spearman correlation of LOXL2 with expression of CTLA-4 in HCC adjusted by purity using TIMER. (d) The expression correlation of LOXL2 with CD274 in HCC determined by GEPIA database. (e) The expression correlation of LOXL2 with PDCD1 in HCC determined by GEPIA database. (f) The expression correlation of LOXL2 with CTLA-4 in HCC determined by GEPIA database.

**Table 1:** Correlation between LOXL2 and different clinicopathological features.

Characteristic	Low-expression of LOXL2	High-expression of LOXL2	p
n	187	187	
Age, n (%)			0.107
≤ 60	80 (21.4%)	97 (26%)	
> 60	106 (28.4%)	90 (24.1%)	
Gender, *n* (%)			0.027
Female	50 (13.4%)	71 (19%)	
Male	137 (36.6%)	116 (31%)	
Race, *n* (%)			0.188
Asian	81 (22.4%)	79 (21.8%)	
Black or African American	12 (3.3%)	5 (1.4%)	
White	88 (24.3%)	97 (26.8%)	
T stage, *n* (%)			0.013
T1	101 (27.2%)	82 (22.1%)	
T2	49 (13.2%)	46 (12.4%)	
T3	33 (8.9%)	47 (12.7%)	
T4	2 (0.5%)	11 (3%)	
N stage, *n* (%)			0.125
N0	121 (46.9%)	133 (51.6%)	
N1	0 (0%)	4 (1.6%)	
M stage, *n* (%)			1.000
M0	130 (47.8%)	138 (50.7%)	
M1	2 (0.7%)	2 (0.7%)	
Pathologic stage, *n* (%)			0.121
Stage I	96 (27.4%)	77 (22%)	
Stage II	44 (12.6%)	43 (12.3%)	
Stage III	34 (9.7%)	51 (14.6%)	
Stage IV	2 (0.6%)	3 (0.9%)	
Histologic grade, *n* (%)			0.029
G1	37 (10%)	18 (4.9%)	
G2	87 (23.6%)	91 (24.7%)	
G3	54 (14.6%)	70 (19%)	
G4	7 (1.9%)	5 (1.4%)	
Tumor status, *n* (%)			0.305
Tumor free	106 (29.9%)	96 (27%)	
With tumor	71 (20%)	82 (23.1%)	

## Data Availability

The original contributions presented in the study are included in the article; further inquiries can be directed to the corresponding author.

## References

[1] Sung H., Ferlay J., Siegel R. L. (2021). Global cancer statistics 2020: GLOBOCAN estimates of incidence and mortality worldwide for 36 cancers in 185 countries. *CA: A Cancer Journal for Clinicians*.

[2] Ferlay J., Colombet M., Soerjomataram I. (2018). Cancer incidence and mortality patterns in Europe: estimates for 40 countries and 25 major cancers in 2018. *European Journal of Cancer*.

[3] Michikawa T., Inoue M., Sawada N. (2015). Plasma isoflavones and risk of primary liver cancer in Japanese women and men with hepatitis virus infection: a nested case-control study. *Cancer Epidemiology, Biomarkers & Prevention*.

The article "LncRNA CARMN Affects Hepatocellular Carcinoma Prognosis by Regulating the miR-192-5p/LOXL2 Axis" was published in 2022. Journal: Oxid Med Cell Longev.

[4] Kimanya M. E., Routledge M. N., Mpolya E., Ezekiel C. N., Shirima C. P., Gong Y. Y. (2021). Estimating the risk of aflatoxin-induced liver cancer in Tanzania based on biomarker data. *PLoS One*.

[5] Lee H. M., Wong W. K. K., Fan B. (2021). Detection of increased serum miR-122-5p and miR-455-3p levels before the clinical diagnosis of liver cancer in people with type 2 diabetes. *Scientific Reports*.

[6] He F., Sha Y., Wang B. (2021). Relationship between alcohol consumption and the risks of liver cancer, esophageal cancer, and gastric cancer in China: meta-analysis based on case-control studies. *Medicine*.

[7] Wen Q., Chan K. H., Shi K. (2022). Tobacco smoking and solid fuels for cooking and risk of liver cancer: a prospective cohort study of 0.5 million Chinese adults. *International Journal of Cancer*.

[8] Triki H., Jeddou H., Boudjema K. (2020). Surgical resection for liver cancer during the COVID-19 outbreak. *Updates in Surgery*.

[9] Niu J., Lin Y., Guo Z., Niu M., Su C. (2016). The epidemiological investigation on the risk factors of hepatocellular carcinoma: a case-control study in Southeast China. *Medicine*.

[10] Zhu Q., Qiao G., Xu C. (2019). Conditional survival in patients with spontaneous tumor rupture of hepatocellular carcinoma after partial hepatectomy: a propensity score matching analysis. *HPB: The Official Journal of the International Hepato Pancreato Biliary Association*.

[11] Cheng Z., Yang P., Qu S. (2015). Risk factors and management for early and late intrahepatic recurrence of solitary hepatocellular carcinoma after curative resection. *HPB: The Official Journal of the International Hepato Pancreato Biliary Association*.

[12] Farhat A., Ferns G. A., Ashrafi K., Arjmand M.-H. (2021). Lysyl oxidase mechanisms to mediate gastrointestinal cancer progression. *Gastrointest Tumors.*.

[13] Wang L., Cao S., Zhai R., Zhao Y., Song G. (2021). Systematic analysis of expression and prognostic values of lysyl oxidase family in gastric cancer. *Frontiers in Genetics*.

[14] Rodriguez-Pascual F., Rosell-Garcia T. (2022). The challenge of determining lysyl oxidase activity: old methods and novel approaches. *Analytical Biochemistry*.

[15] Wang M., Zhao X., Zhu D. (2017). HIF-1*α* promoted vasculogenic mimicry formation in hepatocellular carcinoma through LOXL2 up-regulation in hypoxic tumor microenvironment. *Journal of Experimental & Clinical Cancer Research*.

[16] Lin Z.-Y., Chuang Y.-H., Chuang W.-L. (2012). Cancer-associated fibroblasts up-regulate _CCL2_ , _CCL26_ , _IL6_ and _LOXL2_ genes related to promotion of cancer progression in hepatocellular carcinoma cells. *Biomedicine & Pharmacotherapy*.

The article "LncRNA CARMN Affects Hepatocellular Carcinoma Prognosis by Regulating the miR-192-5p/LOXL2 Axis" was published in 2022. Journal: Oxid Med Cell Longev.

[17] Shao B., Zhao X., Liu T. (2019). LOXL2 promotes vasculogenic mimicry and tumour aggressiveness in hepatocellular carcinoma. *Journal of Cellular and Molecular Medicine*.

[18] Smyth G. K., Michaud J., Scott H. S. (2005). Use of within-array replicate spots for assessing differential expression in microarray experiments. *Bioinformatics*.

[19] Li C., Tang Z., Zhang W., Ye Z., Liu F. (2021). GEPIA2021: integrating multiple deconvolution-based analysis into GEPIA. *Nucleic Acids Research*.

[20] Li J.-H., Liu S., Zhou H., Qu L.-H., Yang J.-H. (2014). starBase v2.0: decoding miRNA-ceRNA, miRNA-ncRNA and protein-RNA interaction networks from large-scale CLIP-Seq data. *Nucleic Acids Research*.

[21] Mousavian Z., Khodabandeh M., Sharifi-Zarchi A., Nadafian A., Mahmoudi A. (2021). StrongestPath: a cytoscape application for protein-protein interaction analysis. *BMC Bioinformatics*.

[22] Liu Y., Khan S., Li L., Ten Hagen T. L. M., Falahati M. (2022). Molecular mechanisms of thyroid cancer: a competing endogenous RNA (ceRNA) point of view. *Biomedicine & Pharmacotherapy*.

[23] Shi Y., Liu J.-B., Deng J. (2021). The role of ceRNA-mediated diagnosis and therapy in hepatocellular carcinoma. *Hereditas*.

[24] Conte F., Fiscon G., Sibilio P., Licursi V., Paci P. (2021). An overview of the computational models dealing with the regulatory ceRNA mechanism and ceRNA deregulation in cancer. *Methods in Molecular Biology*.

[25] Li T., Fu J., Zeng Z. (2020). TIMER2.0 for analysis of tumor-infiltrating immune cells. *Nucleic Acids Research*.

[26] Zhao J., Li L., Guo L. (2021). Nano-gold PCR in detection of TERT methylation and its correlation with hepatitis B-related hepatocellular carcinoma. *Journal of Biomedical Nanotechnology*.

[27] Dong H., Zhang L., Qian Z. (2015). Identification of HBV-MLL4 integration and its molecular basis in Chinese hepatocellular carcinoma. *PLoS One*.

[28] Xu P., Luo A., Xiong C., Ren H., Yan L., Luo Q. (2022). SCUBE3 downregulation modulates hepatocellular carcinoma by inhibiting CCNE1 via TGF*β*/PI3K/AKT/GSK3*β* pathway. *Cancer Cell International*.

[29] AlGabbani Q. (2022). Mutations in TP53 and PIK3CA genes in hepatocellular carcinoma patients are associated with chronic schistosomiasis. *Saudi Journal of Biological Sciences*.

[30] Lin J.-C., Liu T.-P., Andriani V., Athoillah M., Wang C.-Y., Yang P.-M. (2021). Bioinformatics analysis identifies precision treatment with paclitaxel for hepatocellular carcinoma patients harboring mutant TP53 or wild-type CTNNB1 gene. *Journal of Personalized Medicine*.

The article "LncRNA CARMN Affects Hepatocellular Carcinoma Prognosis by Regulating the miR-192-5p/LOXL2 Axis" was published in 2022. Journal: Oxid Med Cell Longev.

[31] Jiang L., Jin H., Gong S. (2022). LncRNA KCNQ1OT1-mediated cervical cancer progression by sponging miR-1270 as a ceRNA of LOXL2 through PI3k/Akt pathway. *The Journal of Obstetrics and Gynaecology Research*.

[32] Li R., Li H., Zhu L. (2021). Reciprocal regulation of LOXL2 and HIF1*α* drives the Warburg effect to support pancreatic cancer aggressiveness. *Cell Death & Disease*.

[33] Zhu G., Wang L., Meng W. (2021). LOXL2-enriched small extracellular vesicles mediate hypoxia-induced premetastatic niche and indicates poor outcome of head and neck cancer. *Theranostics*.

[34] Wu L., Zhang Y., Zhu Y., Cong Q., Xiang Y., Fu L. (2016). The effect of LOXL2 in hepatocellular carcinoma. *Molecular Medicine Reports*.

[35] Wang Y., Ma H., Li Y., Su R. (2022). MiR-192-5p-modified tumor-associated macrophages-derived exosome suppressed endometrial cancer progression through targeting IRAK1/NF-*κ*B signaling. *Reproductive Sciences*.

[36] Gu Y., Ji F., Liu N. (2020). Loss of miR-192-5p initiates a hyperglycolysis and stemness positive feedback in hepatocellular carcinoma. *Journal of Experimental & Clinical Cancer Research*.

[37] Sheng X., Dai H., Du Y. (2021). LncRNA CARMN overexpression promotes prognosis and chemosensitivity of triple negative breast cancer via acting as miR143-3p host gene and inhibiting DNA replication. *Journal of Experimental & Clinical Cancer Research*.

[38] Liu J., Gao M., Yang Z. (2022). Macrophages and metabolic reprograming in the tumor microenvironment. *Frontiers in Oncology*.

[39] Mondello P., Ansell S. M., Nowakowski G. S. (2022). Immune epigenetic crosstalk between malignant B cells and the tumor microenvironment in B cell lymphoma. *Frontiers in Genetics*.

[40] Engelhard V. H., Rodriguez A. B., Mauldin I. S., Woods A. N., Peske J. D., Slingluff C. L. (2018). Immune cell infiltration and tertiary lymphoid structures as determinants of antitumor immunity. *Journal of Immunology*.

